# A Lightweight Deep Learning-Based Approach for Jazz Music Generation in MIDI Format

**DOI:** 10.1155/2022/2140895

**Published:** 2022-08-05

**Authors:** Prasant Singh Yadav, Shadab Khan, Yash Veer Singh, Puneet Garg, Ram Sewak Singh

**Affiliations:** ^1^Department of Computer Science and Engineering, Mahamaya Polytechnic of Information Technology (Govt.), Hathras, Uttar Pradesh 204102, India; ^2^Department of Computer Science & Engineering, Sunder Deep Engineering College, Ghaziabad 201002, Uttar Pradesh, India; ^3^Department of Information Technology, ABES Engineering College, Ghaziabad 201009, Uttar Pradesh, India; ^4^Department of Computer Science, ABES Engineering College, Ghaziabad 201009, Uttar Pradesh, India; ^5^Department of Electronics and Communication, School of Electrical Engineering and Computing, Adama Science and Technology University, Adama, Ethiopia

## Abstract

In today's real-world, estimation of the level of difficulty of the musical is part of very meaningful musical learning. A musical learner cannot learn without a defined precise estimation. This problem is not very basic but it is complicated up to some extent because of the subjectivity of the contents and the scarcity of the data. In this paper, a lightweight model that generates original music content using deep learning along with generating music based on a specific genre is proposed. The paper discusses a lightweight deep learning-based approach for jazz music generation in MIDI format. In this work, the genre of music chosen is Jazz, and the songs selected are classical numbers composed by various artists. All the songs are in MIDI format and there might be differences in the pace or tone of the music. It is prudential to make sure that the chosen datasets that do not have these kinds of differences and are similar to the final output as desired. A model is trained to take in a part of a music file as input and should produce its continuation. The result generated should be similar to the dataset given as the input. Moreover, the proposed model also generates music using a particular instrument.

## 1. Introduction

Music learning is an essential part for the young generation for entertaining life and lives with some happiness. Most schools and even colleges added music subjects across the curriculum by considering the happiness of the students. It develops physiological strong minds along with strong lifelong effects. Practice is the main learning process instead of the theoretical learning process for music. In the initial process of learning, an easy piece of information is required for better understanding the entry-level people.

Music Generation, as the name indicates, means generation of music. This can be achieved either by man creating it or by a computer using various techniques. Machine learning techniques can be used to generate music. There is a new term for the music called Generative music, i.e., popularized by Brian Eno which defines the music, that is, as ever-different and changing created by a system.

We have been acquainted with the concept of machine learning during our time spent developing our knowledge and found that field to be quite interesting. We started exploring different parts of the field, and it further developed our interest in it. It fueled our desire use to apply this concept to solve some real-life problems and we decided to do the same as in this paper. Machine learning is already being used in various fields for further advancements. As technology develops, it has always been our goal to digitalize all tasks and make things easier. However, there are some of the fields where we have not applied the machine learning successfully, but now-a-days, we are able to apply machine learning to perfection in most of the arts like music. Music is one part of the arts in which research is currently being conducted. There is always a constant need for new songs which have to be composed again and again to maintain variety. Using machine learning to solve this problem can be beneficial.

There is a constant demand for new musical content for a multitude of uses, ranging from artistic expression, to jingles for new TV shows, to music in games, and to elevator music. Thus, to train a model by giving it model has to take in a part of a music file as input and should produce its continuation. The result generated should be similar to the dataset given as the input. This proposed lightweight model generates original music content using deep learning along with generating music based on a specific genre. The proposed model also generates music using a particular instrument. The quality of the generated music can be measured by defining some of the measures. In a few algorithms, the outcome can be measured by using their efficiency such as becoming less linear in the case of music generation.

In this paper, the genre of music is Jazz where songs are selected classical numbers composed by various artists. They are collected from various open-source datasets and should be converted into the required MIDI format if they are not already in it. It is prudential to make sure that we choose datasets that do not have these kinds of differences and are similar to the final output we desire. Thus, to train a model by giving it model has to take in a part of a music file as input and should produce its continuation. The result generated should be similar to the dataset given as the input. This proposed lightweight model generates original music content using deep learning along with generating music based on a specific genre.

In this paper, the related work is discussed in Section 2. The system model is discussed in Section 3 whereas Section 4 discusses the proposed methodology. The evolution and analysis of models are explained in Section 5, and finally the paper is concluded in Section 5.

## 2. Related Works

In this section, a study of the existing methods based on the music generations using various machine learning and deep learning models is discussed. Ghatas et al. [1] discuss a hybrid deep learning approach for musical difficulty estimation of piano symbolic music. In this work, a deep convolutional neural network model is trained by using various levels and dividing the roll of the piano. Various features are considered for preparing the models related to handcraft. In this work, a classical music synthesis is performed using recurrent neural network architectures [2], that is, based on the musical scores. This work used two neural network architectures, namely, gated recurrent unit and long-short-term memory for music synthesis. The performance of the models is measured in the form of accuracy and loss. This process also optimizes the input fed during the training process. Dua et al. discuss an approach for sheet music generation that is based on the RNN-LSTM by increasing the accuracy of the music generation [3]. In this work, chord estimation and source separation modules are modified for improvement in the models. This work uses various deep learning models like long-short-term memory (LSTM), and recurrent neural network (RNN) is a hybrid with gated recurrent units (GRUs). Here, the number of sources has separated to increase the accuracy further.

Modrzejewski et al. discuss a method for generating musical phrases using a deep convolutional generative adversarial network [4]. This paper uses classical and jazz music MIDI recordings to train the model. Hsu et al. discuss a new method for generating music transition by using a transformer-based model. The performance of this method is analyzed by using the positive response from listeners. Madaghiele et al. discuss a method for melodic improvisation neural generator using sequence to sequence [5]. Keluskar et al. discuss a method for automatic music generation using deep learning approaches. It uses the sequence of ABC notes for music generation using deep learning like LSTM and GRUs for modeling. In this work, LSTM has worked efficiently. The papers use various machine learning and deep approaches which are used in developing the models in both training and test parts of our models [6–8]. Hewahi et al. discuss a method for pieces of music generation using machine learning where the long-short-term memory neural networks approach is used [9]. This paper uses Bach's musical style for a generation using MIDI files by converting these into song files.

Briot et al. discuss a music generation process using deep learning techniques [10]. This paper discusses the various type of musical content that are generated such as polyphony, melody, and accompaniment. Carnovalini and Roda discuss a multilayered approach to automatic music generation and expressive performance [11]. In this paper, a method is implemented for generating the music for the short massages by the hierarchical structure for the melodies musical contents. This method has checked the performance and analyzed it through the computational method. Dong et al. discuss multi-track sequential generative adversarial networks for symbolic music generation and accompaniment called Musegan [12]. This work uses the generative adversarial networks (GANs) framework for music generation with the help of three models. In the first one, network architecture is discussed, in the second one, the composer model is discussed, and the last one discusses the hybrid model for music generation. The dataset is trained for rock music and applied to generate the piano rolls for the different tracks such as guitar, bass, piano, drums, and strings. Dong and Yang discuss convolutional generative adversarial networks using binary neurons for polyphonic music generation [13]. This process is divided into two phases. In the first phase, the generator and the discriminator are performed. And the second phase network is trained by using the real-valued piano rolls. Nayebi and Gruv discuss algorithmic music generation using recurrent neural networks called Gruv [14]. This method compares the performance of two different models for music generation, namely, LSTM and GRU. The results for LSTM perform better than those for the GRU. In paper [15], jazz transformer-based AI-composed music quantitative measures are discussed. This system measures the jazz transformation using the deep learning model. In paper [16], an analysis-by-synthesis model for jazz improvisation is discussed. In paper [17], a real-time jazz improvisation accompaniment for adaptability of recurrent neural networks is discussed. This is a real-time implementation of the music generation system for jazz improvisation.

## 3. Proposed Methodology

In this section, the methodology of the proposed work is discussed. In the methodology, an essential skeleton structure of the proposed methodology is explained in detail. A basic deep learning model consists of data gathering, data processing, building a model, training the model, and finally using it to generate the result. This work involves the following seven datasets, namely, dataset selection, determination of unique notes, partition into sequences, creation of the model, training of the model, generation of music, and conversion of output to MIDI format as shown in Figure 1.

### 3.1. Dataset Selection

The data to be fed into the model play an important role in the learning process. These data whenever chosen badly might lead to a model that produces bad results. So, even the selection should be done in a careful manner. The data selected should have relevance to the problem statement and context. The initial step involves the selection of songs that are similar in nature meaning that they make use of the same instruments and belong to the same genre. The selection of dissimilar songs results in the generation of unpleasant music. Sometimes, the datasets collected might be from various sources. The care should be taken to modify them into a similar format, i.e., with the same number of features, type of features, same feature values, and feature names.

In this paper, the genre of music is considered Jazz, and the songs selected are classical numbers composed by various artists. All the songs are in MIDI format. They are collected from various open-source datasets and should be converted into the required MIDI format if they are not already in it. Though the genre chosen is Jazz, there might be differences in the pace or tone of the music. It is prudential to make sure that we choose datasets that do not have these kinds of differences and are similar to the final output we desire.

### 3.2. Determination of Unique Notes

The dataset is composed of various songs which increase the number of unique note possibilities that have to be predicted during the process of music generation. Each note to be predicted is analogous to a class in a classification problem of machine learning. In a classification problem, the inputs are taken and manipulated throughout the numerous hidden layers to finally classify them. The number of hidden layers, nodes in each layer, and output layer are all the parameters that are to be decided while before training the model. For this reason, it is essential to know the number of nodes in the output layer, which are equal to the number of classes. So, in this scenario, the number of unique notes is taken as the number of classes. All the music files in the dataset are gone through to gather all the unique notes. These notes are all written to a file for later purposes.

### 3.3. Partition into Sequences

The model takes only a specific number of inputs decided by the model architecture whereas the songs in the dataset might vary in length. This might create a problem in using them as inputs. If the datasets are not fed properly, the results will turn out to be bad. To tackle this problem, the dataset is divided into sequences of equal length which are further used for training the model. These sequences each enter the model as input for one particular instance. The model then trains itself to predict which note is to follow the input sequence. The partition length will be the number of inputs in the model architecture, and hence it is a parameter that is to be carefully chosen.

### 3.4. Model Creating

In this work, the long-short-term memory (LSTM) model is used where the number of layers and nodes in each layer and the hyperparameters are to be tuned to get proper model architecture. There is a cell state in the horizontal line just like a conveyor belt which does not have the facility of adding and removing the information. Gates are used to flow the information as shown in Figure 2 which is composed of various operations like point wise multiplication as shown in Figure 3 and the sigmoid neural net layer. The sigmoid layer outputs consider two binary numbers where zero indicates “let nothing through” and one indicates the “let everything through.” Generally, LSTM consists of three gates that control and protect the cell state [11].

Another approach is dropout which helps in reducing the interdependent learning amongst the various neurons. This method works on the approximation training for a large number of neural networks along with different parallel architectures. In this process, some of the layer outputs are dropped arbitrarily. Dropout makes the training noisy by considering the less responsibility of the inputs. In addition to that, the network layers correct the mistakes. Dropout uses various layers, namely, dense fully connected layers, convolutional layers, and recurrent layers such as the LSTM network layer in a neural network. It drops out a few or all hidden layers in the network [14].

The implementation of various neurons such as LSTM, Dense, Dropout, etc., are done using open-source frameworks for machine learning. There is plenty of machine learning and deep learning frameworks that provide predefined functions that can be used to implement the model architecture. Tensorflow, Keras, Caffe, and PyTorch are a few examples. Considering the ease of use and understanding, Keras has been used in this particular paper [18]. It runs TensorFlow in the backend and provides simple functions to which hyperparameter values can be passed simply for tuning [19].

The model architecture consists of a sequential network. The input layer is connected to the LSTM layer which is then connected to the dropout layer to reduce over-fitting. There can be a series of LSTM layers to increase the feature extraction and functionality of the deep network. The addition of a few dropout layers in between to ensure that the model can learn properly is essential. The final LSTM layer of the model is then flattened into one and is connected to a dense layer to collect all the information from all the nodes into one layer which can now finally be connected to the output layer. The output layer needs an activation function for final computations.

In this stage of the process, an activation function estimates the output of a node in the neural networks given a certain set of inputs. Utilizing the neural networks of the linear perceptron, the activation function of digital networks is accomplished by the use of a chip circuit that is dependent on the binary input. The term “transfer function” can also be used to refer to this function. Tanh, also known as hyperbolic tangent, softmax, threshold or binary step activation function, ReLU, Leaky ReLU, and sigmoid are some of the available forms of activation functions.

The softmax activation function is proven to be very efficient in the case of multiclass classification problems [20]. Sigmoid is mostly used for binary classification. As the number of notes in the songs is always high and is taken as the number of classes too, predicting which note will occur next is also a multiclass classification. So, softmax is used as the activation function in this particular model. Tanh function is also a good choice as an activation function for the problem.

### 3.5. Model Training

The model created is trained using the equal length sequences prepared in the data preprocessing stage. The total dataset which is divided into a number of sequences is run through these sequences to predict the next note to come. The predicted note is compared to the actual note, and loss is calculated. The calculated loss is now used to adjust the different weights and biases in the model such that the next prediction is closer to the actual note next time. This minimizes the loss for the next time.

The same dataset is iterated multiple times. These iterations are generally called epochs which is one of the hyperparameters. Various optimization algorithms such as stochastic gradient descent, Vanilla gradient descent, batch gradient descent, and Adam optimizer can be used for adjusting the weights. Each has its own advantages and disadvantages which makes the choice tough but important.

The main goal of training the model repeatedly through the epochs on the same dataset several times is to reduce the loss of the model while increasing the probability of predicting the next node with a better choice than the last time. The number of epochs, size of the dataset, batch size, number of hidden layers, and their nodes are all hyperparameters that are to be tuned, i.e., different combinations of all of them are to be tried and each of them has to be adjusted based on the previous results in order to obtain better results the next time.

### 3.6. Generation of Music

Now, a music file that is similar to the desired output is taken and converted into MIDI format if not already of that type and then sent through the data preprocessing phase and sent as an input to the trained model which then predicts the further notes until a predefined length. The initial part of the file, which is of the same length as the partitioned sequences (i.e., size of the input), is passed as the input to the model. The model then predicts the next note which is appended to the input. The first note of the new input is now discarded to maintain its length. This input is fed again to the model for the prediction of the second note, following the first note.

Repeating the steps of adding the new note that was predicted while throwing away the previous piece in order to keep the same size will continue to be done until the appropriate length has been determined. As part of the process of producing the output, each of the predicted notes is attached to the initial partition. The collected output is now written into a file that is being saved in order to make it available for access whenever it may be required. A continuous stream of sounds and chords has been produced as the output at this point. Due to the fact that they are still in their numerical format, they cannot be played for a person to listen to and appreciate.

### 3.7. Conversion of Output to MIDI Format

The obtained output from the file is taken and is to be converted into MIDI format. In music generation, the output cannot be directly evaluated as it is not a value that can be compared and checked for accuracy. The music is to be heard to judge if the generated music produces the desired music in the right genre with the right instruments and most importantly if it is good to hear. In order to do this, the output file is converted back to MIDI format with the help of open-source libraries or online converters. This output can now be played using a music player and can be transferred and enjoyed just like any other music file. The MIDI file can also be converted to other formats such as MP3, WAV, and OPUS, using converters if at all necessary.

## 4. Evolution and Analysis of Models

The music derives meaning through repetition and modeling musical coherence created by internal repetition, and reference to earlier material in a piece is a persistent issue in computational music generation and presents a challenge, especially when creating a model. The generation of music is a problem in which the outputs cannot be graded quantitatively. Hence, metrics like accuracy, precision, or recall lose their relevance. The evaluation of the model can be conducted based on either being graded by humans or through the effectiveness of the loss function. The loss function of the model in the initial stages of the training is observed. It gradually decreases throughout the multiple iterations of the learning phase. If the loss is optimized to the desired extent and the output generated by the model is considered to be satisfactory, then the model is said to be performing well. Hence, the loss value in the final iterations/epochs of the training should be at an optimum value. The model is trained using two-piano MIDI datasets. In this work, the deep jazz dataset is used for checking the performance of the proposed model. The classical dataset is taken for the MIDI file [20]. The datasets are further classified as firstly, the dataset contains 20 minutes of music while the second dataset contains approximately 50 minutes of music.  Figure 4 shows the proposed model results for different datasets, i.e., midi files dataset 1, midi files dataset 2, classical dataset by considering the dataset length in minutes, the number of epochs runs, time for each epoch in seconds, batch size, initial loss value, and final loss value. Also, Table 1 shows the results analysis of the model for different datasets.

The same model has been trained with a new dataset that contains classical piano music for 10 minutes in total. The model still works well and obtains an optimum loss value and also generates good classical piano music. The proposed model can be used to generate new content depending on the dataset that has been provided. Since the individual's preferences serve as the basis for both the input and the training dataset and since the music that is produced by the music is similar to the datasets that are used, any newly generated songs will also be similar to the datasets, which will further increase the likelihood that the user will enjoy listening to them. The same concept that is utilized in the process of generating music can also be utilized in the process of converting text-to-speech. The notes that are provided as input are processed by the music generation model, which then makes predictions about the notes that will come next. In the same vein, the format of the alphabets in the text can be thought of as being comparable to that of the numbers in the notes. In the same way that the numerical forms can be converted back to MIDI and played as live music, the transformed characters can make phonetic sounds where speech would normally be. Therefore, the model may be trained using more accurate datasets and more powerful GPUs to create a text-to-speech model as well. Also, Table 2 shows the results analysis of the model for loss with respect to the epoch.

Figure 5 shows the proposed model results for the loss vs. epoch for different datasets, that is, midi files dataset 1, midi files dataset 2, and classical dataset. It is evident from Figure 5 that as the number of epochs are increased the loss value decreases. The loss value at the 10 epoch is 4.12, 4.56, and 2.60 for midi files dataset 1, midi files dataset 2, and classical dataset, respectively. In the mid of the epochs when the value of its 50, the loss value is 0.39, 0.34, and 0.11 for midi files dataset 1, midi files dataset 2, and classical dataset, respectively. The loss value at the 100 epoch is 0.03, 0.06, and 0.01 for midi files dataset 1, midi files dataset 2, and classical dataset, respectively.

## 5. Conclusion

In this paper, a lightweight deep learning-based approach for jazz music generation in MIDI format is proposed. This system can be utilized for generating music in a specific genre, played with a particular instrument. The weights of the trained model can be saved and loaded when required. This eliminates the enormous amount of time wasted on training the model again and again. The music generated can be used to fulfill various demands in several industries. The paper has been conducted in a system environment that is not capable of performing large calculations in a small amount of time. This limits the size of the dataset that can be used for learning thereby causing the model to underperform in certain cases. Provided with a GPU with a high computational performance enables us to use bigger datasets and also reduces the time of training the model, thereby producing far better results in a very less amount of time. The model can also be used for creating personalized music for an individual. The songs liked by the user and belonging to a particular genre can be all used as the dataset to train the model. The model can then be used to generate fresh content based on the provided dataset. As the input and the training dataset are based on the favorites of the individual and the music generated by the music is similar to the datasets used, the further newly generated songs will also be similar to the datasets which further increases the chance of the user liking them. The model used for generating music can also be used for text-to-speech conversion. The music generation model uses the given input notes and predicts the following notes. In the same way, the alphabets in the text can be considered analogous to the numeric format of the notes. Just as the numeric formats when converted back to MIDI and played live music, the characters when converted produce phonetic sounds where speech is. Hence, the model can be trained with better datasets and GPUs to build a text-to-speech model too [21–25].

## Figures and Tables

**Figure 1:** Block diagram of the proposed methodology.

**Figure 2:** LSTM gates [16].

**Figure 3:** LSTM multiplication operation [18].

**Figure 4:** Proposed model results for different datasets.

**Figure 5:** Proposed model results for the loss vs. epoch for different datasets.

**Table 1:** Results analysis of the model for different datasets.

Data set	Midi files dataset 1	Midi files dataset 2	Classical dataset
Dataset length	20 minutes	50 minutes	20 minutes
Number of epochs run	100	100	50
Time for each epoch	∼26 seconds	∼62 seconds	∼35 seconds
Batch size	16	16	16
Initial loss value	4.88	4.88	4.69
Final loss value	0.031	0.062	0.117

**Table 2:** Results analysis of the model for loss with respect to the epoch.

Number of epoch	Midi files dataset 1	Midi files dataset 2	Classical dataset
**10**	4.12	4.56	2.60
**20**	2.34	2.89	0.92
**30**	0.84	0.64	0.52
**40**	0.40	0.41	0.41
**50**	0.39	0.34	0.11
**60**	0.38	0.24	0.10
**70**	0.18	0.24	0.02
**80**	0.04	0.22	0.02
**90**	0.04	0.20	0.01
**100**	0.03	0.06	0.01

## Data Availability

Data will be available on request to Yash Veer Singh (yashveersingh85@gmail.com).
